The article "Dimensional Analysis of Regional Environmental Planning Based on NPP/VIIRS Lighting Data" was published in 2022. Journal: Comput Intell Neurosci.

# Dimensional Analysis of Regional Environmental Planning Based on NPP/VIIRS Lighting Data

**DOI:** 10.1155/2022/4132904

**Published:** 2022-08-09

**Authors:** Haizhang Yan

**Affiliations:** School of Computer Science and Technology, Xidian University, Xi'an 71000, China

## Abstract

The actual status of the current regional environmental planning is difficult to obtain through traditional statistical methods, and it is necessary to use remote-sensing identification technology to collect information. Based on the NPP/VIIRS technology, this study uses the NPP/VIIRS technology to identify and analyze China's regional environment. Moreover, on this basis, this study conducts a dimensional analysis of regional environmental planning, verifies the feasibility of the technology, and promotes the development of the technology in environmental planning. In addition, this study links light intensity and carbon emissions based on night-light data and traditional energy consumption data. Finally, from the perspective of time and space continuity, new solutions and research methods are provided for many problems existing in traditional carbon emission research, which in turn provides a solid scientific foundation and theoretical basis for the formulation and implementation of carbon emission reduction strategies. The research results show that the method proposed in this study has certain effects.

## 1. Introduction

Since the reform and opening up, with the acceleration of China's industrialization process, science and technology and social productivity have greatly improved, and China's economy has shown a sustained and rapid growth trend. However, while the overall national strength has steadily increased and the people's quality of life has been continuously improved, the consumption of natural resources and the discharge of pollutants have also significantly increased, which has worsened the ecological environment and increased the conflict between economic development and environmental pollution [1].

With the rapid development of society and economy, environmental issues have become increasingly prominent. Since the 1960s, environmental disasters have been common in the world, which not only harm the environment itself and human survival, but also have become an important factor restricting social and economic development. The global risk report divides the global risk system into five parts: economic risk, environmental risk, geopolitical risk, social risk, and technical risk. The report analyzes and comprehensively evaluates the statistical data of various regions around the world over the years. It is pointed out that Asian countries have the fastest urbanization process, and their environmental risks are more serious than other continents and regions. In China, as the level of modernization continues to increase, areas with high population and enterprise clusters have gradually increased. This trend provides favorable conditions for better organization of production and strengthening of links and division of labor in various industries in the region, and promotes rapid development of the regional economy and industry, but at the same time, it also brings major hidden dangers to society. The number of risk sources in the region is large and dense, and dangerous substances such as flammable, explosive, poisonous, and harmful are concentrated in large quantities. Once an accident occurs, it will lead to large-scale damage and may also cause the domino effect of the accident, which will not only cause huge property losses, and endanger the health of the people, but also directly affect regional economic development and social stability.

In China, the characteristics of air pollution are compound pollution. At the same time, the sustained development of regional economy and society in China and the concentrated discharge of atmospheric pollutants have made regional air pollution characteristics appear more and more frequently in China [2], and the frequency of severely polluted weather has increased in neighboring cities in the region. Facing the severe environmental situation, China has made relevant requirements for local governments in the “Air Pollution Prevention Action Plan”: local governments need to incorporate severely polluted weather into the emergency management of local governments, and take timely measures to limit production, emissions, and motor vehicles of heavy polluting enterprises according to pollution levels. Years of meteorological data and air quality statistics in the region are the basis for establishing an air pollution emergency plan. In addition, years of meteorological data provide a basis for judging the weather situation causing heavy pollution, and air quality monitoring provides basic data for emergency plans and provides a basis for determining the conditions for starting emergency plans. The construction of ambient air quality monitoring stations can provide monitoring data for the environmental emergency warning system, and also provide a basis for formulating air pollution control plans and proposing preventive measures. Therefore, the deployment of urban air quality monitoring points is of great significance.

The deployment of ambient air quality monitoring points requires comprehensive consideration of various factors. Relevant researchers have carried out a lot of work in order to maximize the overall benefits of the environment, economy, and society, and set up as few monitoring points as possible to reflect the ambient air quality in the monitoring area. These studies mainly focus on the improvement of existing monitoring networks, but relatively few studies have been conducted on setting up monitoring points in newly developed areas or areas lacking monitoring data [3].

Based on the NPP/VIIRS technology, this study uses the NPP/VIIRS technology to identify and analyze China's regional environment. Moreover, on this basis, a dimensional analysis of regional environmental planning is performed to verify the feasibility of the technology and promote the development of the technology in environmental planning.

## 2. Related Work

In view of the current status of China's regional environment and combined with the needs of sustainable development, a more effective carbon emission reduction policy should be adopted [4]. Yang et al. carried out urban development monitoring and evaluation based on night-light data [5]. Luxia proposed that DMSP/OLS night-light images have the potential to extract urban built-up areas [6]. However, the application of early DMSP/OLS night-light data was limited by many factors such as pixel saturation, light overflow, cloud cover, and transient light sources. How to reduce and eliminate these limiting factors has been accompanied by the development of the application of DMSP/OLS night-light data [7]. Later, based on the DMSP/OLS data, Zheng [8], Kellner [9], Chen [10], Lin [11], Favorskaya [12], and others have monitored and analyzed the spatial expansion of cities in different regions and at different scales.

Yinjiang constructed a light index based on the DMSP/OLS nonradiation calibration night-light average-intensity data, proving that the light index can be used for the assessment and monitoring of urbanization levels and processes [13]. Hu et al. [14] further constructed a light index (CNLI) with a certain physical significance and studied the spatial-temporal characteristics of China's provincial urbanization level. Dev et al. [15] used DMSP/OLS night-light data to extract the urban information of the Bohai Rim region in the 1990s, analyzed its urbanization process, and further combined the statistical data to reconstruct the urbanization spatial process of mainland China in the 1990s. Shiming combined the lighting data and the gravity model to measure and divide the hierarchical structure and spatial pattern of China's urban system [16]. Liao et al. [17] carried out a series of studies on urbanization issues such as land urbanization level, urban agglomeration size distribution, and urban land-use and population size distribution based on DMSP/OLS night-light data in the Bohai Rim region. Morley [18] and Zhang [19] extracted urban land from night-light data of Jiangsu Province, Yangtze River Delta, Zhejiang Province, and Bohai Rim, respectively, and analyzed and discussed issues related to urbanization in specific regions.

At present, foreign CO_2_ emission measurement methods mainly include research methods such as the material balance algorithm, emission coefficient method, model method, and life cycle method. However, as far as the actual domestic research situation is concerned, the calculation method based on detailed fuel classification provided by IPCC (2006) is mainly used [20]. Wang et al. estimated the amount of CO_2_ emitted into the atmosphere by global fossil fuel consumption and cement production in the 1980s based on detailed fuel inventory data, accounting for approximately 78% of anthropogenic carbon emissions [21]. Han Y et al. decomposed the influencing factors of carbon emissions into population number, GDP per capita, energy intensity, and energy structure, and constructed the famous Kaya identity, which has been widely recognized and applied [22]. Lu et al. applied the adaptive weighted division method to the decomposition of manufacturing carbon emissions in one country. Moreover, they found that the reduction in energy intensity, that is, the increase in average factor productivity, caused the decline in total carbon emission intensity in these countries to range from 30% to 70% [23]. Based on the national data of two or three sectors with international industrial standards, Hui-Ping et al. used the adaptive weighted Dirichlet decomposition method to analyze the evolution of carbon emissions in manufacturing sectors in 13 IEA countries. Moreover, they also explained the impact of energy intensity and mixed fuel energy on carbon emission intensity [24]. Gao et al. clarified the scope of application of the STIRPAT model and ecological resilience. By calculating the CO_2_ and energy footprint generated by the burning of fossil fuels, they studied the interrelationship between carbon emissions and energy consumption and population and economy [25]. Zhang et al. used a modified Laspeyres model to decompose Greek carbon dioxide emissions and followed a bottom-up approach to explain the reasons for the increase in observed CO_2_ emissions. In order to follow the objectives of the Kyoto Protocol, they proposed a policy priority [26]. Aiming at the respective carbon emission reduction targets of China and India, namely, to reduce 40–45% and 20–25%, respectively, Jiao et al. used a stochastic frontier model to predict the carbon emission intensity of the two countries. The results show that China's target setting requires potential conditions compared to India, including measures such as biofuels and hybrid vehicles. It is concluded that human beings face difficulties in finding sustainable, low-carbon, and cost-competitive petroleum fuel alternatives, and there is a long way to go to reduce greenhouse gas emissions [27].

## 3. Luminous Remote-Sensing Technology

In the absence of clouds at night, the process by which remote-sensing sensors acquire visible light sources on the ground is called luminous remote sensing. Luminous remote sensing originated from DMSP/OLS, and it was originally designed to capture the weak reflection of moonlight on the moon at night, and then, obtain the distribution information of the cloud at night. However, in actual applications, it was found that DMSP/OLS can also capture the light information of the ground under cloudless conditions, thus opening the door to the development of luminous remote sensing. At present, luminous remote-sensing data sources are relatively abundant. The luminous remote-sensing images that can be obtained for free mainly include DMSP/OLS images and NPP/VIIRS images. Argentina and Israel also have their own spaceborne low-light detection instruments, but due to lack of data, they have not been widely used. In the future, the United States will continue to launch related satellites equipped with VIIRS. China will also launch a self-developed “Lujia-1” scientific experimental satellite in the near future, equipped with luminous remote-sensing cameras and navigation enhancement loads, to obtain luminous remote-sensing data, and carry out experimental applications of low-orbit luminous remote sensing.

The DNB/SDR night-light image is a secondary image product after system geometric correction. To further improve the image quality, it is necessary to perform geometric fine correction on the original SDR image. The research is based on ENVI 5.3 software and uses the polynomial method to perform geometric fine correction on the original SDR image. The principle is to establish a polynomial spatial transformation and pixel difference calculation between different images through several control points to achieve the registration between the remote-sensing image and the geographic image, so as to reduce or eliminate the geometric distortion of the image. The original radiation unit of DNB/SDR data is W/(sr·cm2) W/cm^2^/sr, and its original radiation value is usually between 10^−11^ and 10^−8^ W/(sr·cm^2^). Moreover, there are usually 7 to 10 zeros after the decimal point and before the effective radiation value. Too small radiation value will cause inconvenience to both data reading and processing. Therefore, the original radiation value is uniformly multiplied by 10^9^ to convert its radiation unit to nW/(sr·cm^2^), and the corresponding radiation value is also converted to 10^−2^ nW/(sr·cm^2^) or more. The VIIRS/DNB is vulnerable to white noise due to changes in scanning angle during scanning imaging, and the noise level at the edge of the scanning band is higher than the subsatellite point. This research uses the Wiener filter to filter and reduce the noise of DNB image. Wiener filter is an adaptive filter that calculates the mean square error of the radiation values in a 3 ×  3 neighborhood in the image and implements the optimal filtering based on the minimum mean square error criterion, which has a good filtering effect on white noise.

In order to obtain the characteristic light radiation information, the radiation difference between the light and the background pixels should be enlarged as much as possible. The spike median index (SMI) proposed by Elvidge was used to amplify the difference in radiation between the light and background pixels.

First, a 3  ×  3 median filter is used to smooth the preprocessed image. Median filtering is to take each pixel in the image in its neighborhood to take the intermediate brightness value instead of the pixel value, so as to remove the “bright spots” in the image while keeping the original image information as much as possible. Then, by making a difference between the median filtered image and the preprocessed image, the difference between the “bright spots” and the background pixels in the image can be further enlarged to obtain a characteristic image of the light (Figure 1).

For images with large differences in radiation between the target and background pixels, threshold segmentation is an effective image segmentation method, and threshold selection is the key to threshold segmentation. The accuracy of threshold selection is directly related to the effect of threshold segmentation. In this study, the maximum entropy method (MaxEnt) was used to perform adaptive threshold segmentation on the light feature image. In information theory, entropy is a measure of the uncertainty of random variables. If the pixel radiation value of a digital image is regarded as a set of random variables, then the entropy of the image is a characteristic parameter that measures the randomness of the radiation level distribution. In the process of image segmentation, the closer to the boundary between the target and the background, the greater the uncertainty (entropy) of its classification. The maximum entropy threshold segmentation is based on the above assumption, that is, during the segmentation process, the sum of the entropy values of the target and the background should be maximized. Compared with fixed threshold segmentation, maximum entropy threshold segmentation has a better segmentation effect and adaptability. The maximum entropy threshold segmentation effect is shown in Figure 2. The segmentation result is output in the form of a CSV file for subsequent analysis and processing. The formula for calculating the maximum entropy threshold is as follows:

(1) $$\begin{array}{c} {\text{Thr}}_{\text{ent}}=\text{argmax}\left(H\right)\\ =H_{F}+H_{B}\\ =\left(-\sum_{X=\text{min}\left(\text{Rad}\right)}^{Thr}p\left(x\right)\log\;p\left(x\right)\right)+\left(\sum_{X=\mathrm{Thr}}^{\text{max}\left(\text{Rad}\right)}p\left(x\right)\log\;p\left(x\right)\right). \end{array}$$

In the formula, Thr is the abbreviation of threshold (Threshold); *Thr*_ent_ is the maximum entropy threshold; *H* is the sum of the entropy of the target *H*_*F*_; the background *H*_*B*_ is the pixel radiation value; *p*(*x*) is the probability of the pixel radiation value in the histogram; min(Rad) is the minimum pixel radiation value in the image; and max(Rad) is the maximum pixel radiation value in the image.

The maximum entropy method can achieve the optimal threshold segmentation between “bright spots” in the image and background pixels, but not all “bright spots” in the actual situation are lights. The spatial resolution of the DNB image is 742 m. The higher power of the light may cause its neighboring pixels to be illuminated, which will also appear as “bright spots” with high radiation values on the DNB image and be mistakenly recognized as lights in the threshold segmentation. The essence of the local spike detection, LSD, algorithm is to start from the spatial close relationship between the “bright spots” in the maximum entropy threshold segmentation result and find and remove these nonlight “bright spots” to accurately extract the lights from the image (Figure 3). The implementation steps of the LSD algorithm are as follows:

1. In the maximum entropy threshold segmentation result, the first row of pixels is defined as pixel *i*, and the remaining pixels are, respectively, defined as pixels j1, j2, j3,…, jn, and the spatial distance between pixels *i* and *j* is calculated.
2. The spatial resolution of the DNB image is 742 m. If the distance between *i* and *j* does not exceed 742 m, it indicates that the pixel is *i*, j is a neighboring pixel, and its energy gradually decreases with the increase in distance during the light propagation process. Therefore, the pixel with the larger SMI value in the two pixels is defined as the pixel *i*, and the cycle is repeated until the pixel with a distance of less than 742 m from the pixel *i* is not found, and the last pixel *i* is output as a1. At the same time, it is deleted from the original CSV file.
3. After completing the process of outputting cell a1, the first row of cells in the remaining cells of the CSV file is defined as cell *i*, and step (2) is repeated until all cells in the CSV file are deleted. The corresponding output result is the position and brightness information of the pixel where the light is located. Green in Figure 3(b)) is the local unique light extracted by the local peak detection algorithm.

The VMS is a comprehensive application system integrating global satellite positioning, electronic maps, electronic charts, computer network communications, and database technologies. Its main function is to obtain and store the ship's position and operating status information in real time and transmit this information to the monitoring center through network communication to realize the information interaction between the monitoring centers. VMS can record dynamic information in real time, its return frequency is 4 h, and its positioning accuracy is 10 m. The position of the light remains basically unchanged, so the position of the same operation light reflected on the DNB image and VMS data within 4 h is basically unchanged. Because the VMS data do not contain status information, it is necessary to remove the nonoperational VMS data through the light MS data extraction algorithm before verification. If the position of a VMS data record in a certain period is located in the buffer, the light corresponding to the VMS data can be considered to be in the operating state (the VMS ship position in the operating ocean light buffer in Figure 4 is the extracted position).

## 4. Data Source and Preprocessing

Based on the night-light data and energy consumption data, carbon emission simulation was performed. First, the ArcGIS zonal spatial analysis tool was used to statistically study the total value of the light DN in the area, and the curve change diagram is shown in Figure 5. It can be seen that the total value of DN of image pixels in the study area shows a regular year-by-year increasing trend. Second, based on detailed energy statistics, the IPCC carbon emission inventory method is used to measure the carbon emission in the area, and the carbon emission curve is plotted, as shown in Figure 6. It is found through comparison that both the carbon emission measurement value and the total value of the light image pixel DN are increasing year by year and show consistency in time series. Furthermore, the correlation coefficient between the total value of the light pixel DN and the carbon emission is calculated (Figure 7). It can be seen that, regardless of the overall or provincial units, the correlation coefficient between the two is high. The revised regional correlation coefficients of the “potential lighting area” were 0.91, 0.95, 0.98, 0.99, 0.97, and 0.98 (the study area), all showing a high correlation. After the “potential light area” treatment, the correlation coefficient and correlation of the two have been effectively improved to varying degrees. The above comparison and analysis further indicate that there is a certain connection between night-light images and carbon emissions of energy consumption, and further verify the appropriateness, rationality, and scientificity of using night-light data to simulate energy consumption carbon emissions.

## 5. Dimensional Analysis of Regional Environmental Carbon Emissions

From 1999 to 2019, the carbon emissions in the studied areas have been increasing. The carbon emissions in 1999 were 61338.05 million tons; the carbon emissions in 2002 were 1189.8873 million tons; the carbon emissions in 2007 were 14.109872 million tons; the carbon emissions in 2012 were 22.346657 million tons; the carbon emissions in 2017 were 2,96,178,780 tons; and the carbon emissions in 2019 were 3,162,280,800 tons. The average growth rate of carbon emissions from 1999 to 2003 was 11.36%, and the increase was 511.0258 million tons. The growth rate of carbon emissions from 2007 to 2009 has slowed down; the average growth rate is 5.32%; and the increase is 42908846 tons. The growth rate of carbon emissions from 2010 to 2017 has increased compared with the previous stage; the average growth rate is 7.27%; and the increase is 77.172 million tons. From 2015 to 2019, the emission reduction effect has been obvious in recent years; the growth rate of carbon emissions has been significantly reduced compared to the previous stage; and it is also the slowest of the four stages, with an average growth rate of 3% and an increase of 474.387 million tons.

As shown in Figure 8, from 1999 to 2019, as a whole, the trend of high carbon emissions in the Ring region and low carbon emissions in the north and south can be divided into five stages. From 2004 to 2006, the carbon emissions in the studied regions were generally low; Region 4 was the highest, and Region 4 cities were the carbon emission centers in the Ring 6 region. From 1998 to 2000, the other regions in the Ring 6 region were low-carbon-emission regions. The overall pattern of carbon emissions in the Ring 6 region was not yet known. From 2001 to 2006, the pattern of high carbon emissions in the Ring region and low levels in the Ring and southern regions of the Ring 6 region began to form. On the whole, the carbon emissions in the Ring region were high, and the carbon emissions in the north and south were low. In addition to the high-value areas such as Regions 4 and 5, the Ring areas of the Ring 6 region, that is, the south of the Region 3 province, the east of the Region 1 province, and the south of the Region 2 province, have also changed from a low-carbon-emission region to a stable high-value region, which includes some cities in Region 3 province, Region 1 province, and Region 2 province. At this stage, Regions 4 and 5 have gradually become the carbon emission centers of the Ring 6 regions. The carbon emission centers in the Ring 6 region have expanded. The low-carbon-emission areas in the north of the Ring 6 region have remained stable, and the low-carbon-emission areas in the south of the Ring 6 region have a tendency to transition to high-value regions. From 2007 to 2009, some regions in the Ring 6 region began to transform into carbon emission centers. The pattern of high carbon emissions in the middle and low in the north and south of the Ring 6 region has not changed. Regions 4 and 5 remain the carbon emission centers of the 6th region. The southern regions of Region 3 province, the eastern regions of Region 1 province, and the southern regions of Region 2 province have a tendency to transform into regional carbon emission centers. The low-carbon-emission value in the northern part of the Ring 6 region remained stable, and the southern part of the region turned into a high-value region. From 2010 to 2017, some regions in the Ring 6 region formed a carbon emission center stage. Beginning in 2010, the carbon emission centers in the Ring 6 region are no longer just Region 4 and Region 5 cities. The single center of carbon emissions in the Ring 6 region has become a multicenter, forming the largest carbon emission center in the Ring 6 region. A large-scale carbon emission center has also been formed in the eastern part of Region 1 province, and the remaining three individual prefecture-level carbon emission centers have also been formed in the Ring 6 region. Only some prefecture-level units in the northern part of the Ring 6 region have a tendency to evolve to high-value areas, and the low-value areas in some parts of the south continue to shift to high-value areas. From 2018 to 2019, carbon emissions in the Ring 6 region have risen as a whole, and some regions have decreased. Several carbon emission centers in the Ring 6 area remain stable. There are still two large regional carbon emission centers and three single centers. The most obvious difference between this stage and the previous stage is that, first, as a whole, the carbon emissions in the Ring 6 region are generally from a low value to a high value. This is a clear phenomenon that the carbon emissions in the Ring 6 region generally rise. Second, the carbon emissions of some high-value centers have begun to decline, which is a signal of carbon emission reduction in some regions. In general, the carbon emissions in the Ring 6 region show a steady state of high in the middle and low in the north and south. Multiple carbon emission centers have gradually formed in some areas of the Ring 6 region. The carbon emissions in the area of the Ring 6 region have increased continuously over time and gradually changed from low-value areas to high-value areas. At the same time, in the past two years, some regions in the Ring 6 region also have a tendency to reduce carbon emissions. This is due to the implementation of emission reduction policies.

In terms of the spatial distribution of per capita carbon emission intensity (Figure 9), the per capita carbon emission intensity of the prefecture-level research units in the Ring 6 region was relatively low in 2000, and the low-value regions were located around the entire Ring 6 region. In 2005, the per capita carbon emission intensity of the Ring 6 region significantly increased, and many regions changed from low-value to high-value areas. In 2010, the per capita carbon emission intensity of the Ring 6 region has increased to a certain extent on the basis of 2005, and the distribution of high-value regions has become more obvious on the basis of 2005. The area along the Jiqing line in Region 1 forms a high-value area, and the low-value area is further reduced. In terms of the intensity of carbon emissions per unit of GDP (Figure 10), in 2000, the intensity of carbon emissions per unit of GDP of prefecture-level research units in the Ring 6 region was relatively high, especially in the west and north of Region 2, forming a continuous high-value area. In 2005, the intensity of carbon emissions per unit of GDP in the prefecture-level research units in the Ring 6 region decreased compared with 2000. The area along the Beijing-Shenzhen line formed a large area of high-value distribution, and a large area of low-value distribution was formed throughout the entire Region 1 province. In 2010, the intensity of carbon emissions per unit of GDP of the prefecture-level research units in the Ring 6 region significantly dropped, and it was distributed in a “C” shape throughout the Ring 6 region.

## 6. Analysis and Discussion

This study has performed a series of processing and correction on night-light data and put forward the concept of “potential light area” to quickly extract valid light information in a specific range. Moreover, this study combines the energy consumption data of each province (city) to ideally simulate the regional carbon emissions. Through downscaling research methods, carbon emissions at multiple scales such as provincial, prefecture, and county levels have been more reliably simulated and analyzed. Moreover, this study analyzes the time-series changes, spatial-temporal distribution characteristics, and spatial pattern evolution of carbon emissions at various scales. In addition, the geographic detector software was used to reveal the impact mechanism of carbon emissions in the region, which provided a scientific basis and theoretical basis for the formulation of refined and differentiated regional carbon emission reduction strategies.

In this study, the processing procedures of relative radiation correction, intrayear synthesis correction, and interannual sequence correction are performed on the stable-light data, which better solves the problem of pixel saturation in the central area of the city, the pixel difference of different satellites in the same year, and the abnormal fluctuation of the same satellite in different years, and makes the night-light pixel DN value more in line with the actual situation in the region. Based on the night-light data of NPP/VIIRS, the concept of “potential light area” was proposed, which effectively reduced the problem of a large number of low-value pixels in nonlight source areas; the correlation coefficient between the DN value of light pixels and carbon emissions was improved; and the simulation was more in line with the actual situation.

Studies have shown that the cycle of carbon is always one of the basic factors and sources of power that determine global climate and environmental change. With the rapid expansion of the material and energy exchange scale of the terrestrial surface system and the continuous acceleration of the exchange rate, the asymmetric development of the carbon cycle (more emissions and less absorption) is showing more and more negative effects on the global environment, especially on climate change. Therefore, it has become a focus of common concern of scientists from all over the world. With the rapid development of the economy and society, the greenhouse gases emitted by large-scale human activities (such as the use of fossil fuels, cement production, and land-use change) have deeply disrupted the carbon cycle of nature. Among them, CO_2_ emissions from energy consumption using large-scale fossil fuels account for as much as 60% of total greenhouse gas emissions, which is the primary contributor to climate warming. Therefore, studying the CO_2_ emissions caused by human activities (especially energy consumption) has become a hot issue in academic circles at home and abroad. Carbon trading, carbon emission reduction, and carbon decoupling have become important policy measures to mitigate global warming.

The “potential lighting area” proposed in this study largely meets the need to quickly and efficiently extract the effective pixels in the research area. However, the threshold setting should take into account the different levels and development levels of cities to set the level, classification, and local errors that may be caused by a single threshold. Even so, the actual situation can be better approximated only by accurately extracting the effective construction land range in the light image. However, considering the trade-off between time and efficiency, here, unlike monitoring urban expansion, precise construction land extraction is required. Therefore, this study does not set the threshold year by year or use other methods to extract construction land, but only counts the total value of the light pixel DN in a specific area (i.e., “potential light area”). Practice has proved that this method achieves better results in carbon emission simulation and can meet the basic needs of this study.

## 7. Conclusions

Since the 1970s and 1980s, night-light images have been widely used in many research fields such as urban monitoring and evaluation, socioeconomic parameter estimation, and major event evaluation, which provide a unique perspective and strong support for capturing and understanding human activities at night. Because carbon emissions are closely related to human economic activities, and economic activities have a strong correlation with luminous light, luminous light can be used to reflect the spatial distribution of carbon emissions and spatialize carbon emissions. Based on night-light data and traditional energy consumption data, this study links the light intensity with carbon emissions, provides new solutions and research methods for the abovementioned problems in traditional carbon emission research from the perspective of continuous time and space, and then provides a solid scientific foundation and theoretical basis for the formulation and implementation of carbon emission reduction strategies. At the same time, this study further enriches the breadth and depth of the research content of night-light data.

## Figures and Tables

**Figure 1:** (a) Wiener filtering effect. (b) Median filtering effect. (c) Peak median exponential effect.

**Figure 2:** Median peak value index of pixels based on maximum entropy threshold segmentation.

**Figure 3:** Example of the effect of the local peak detection algorithm. (a) Maximum entropy threshold segmentation effect. (b) Local peak detection effect.

**Figure 4:** Extraction effect of VMS data of working lights.

**Figure 5:** Trend of the total value of DN of the lighting pixel.

**Figure 6:** Trend of carbon emission measurement.

**Figure 7:** Correlation coefficient between the total value of DN of light pixels and carbon emissions in the study area and provincial administrative units.

**Figure 8:** Spatial distribution of carbon emissions at scale.

**Figure 9:** Spatial distribution of per capita carbon emission intensity.

**Figure 10:** Spatial distribution of carbon emission intensity per unit of GDP.

## Data Availability

The data in this article can be obtained from the author upon request.
